# Prediction of Heart Disease Using a Combination of Machine Learning and Deep Learning

**DOI:** 10.1155/2021/8387680

**Published:** 2021-07-01

**Authors:** Rohit Bharti, Aditya Khamparia, Mohammad Shabaz, Gaurav Dhiman, Sagar Pande, Parneet Singh

**Affiliations:** ^1^School of Computer Science and Engineering, Lovely Professional University, Phagwara, India; ^2^Department of Computer Science, Babasaheb Bhimrao Ambedkar University, Lucknow, India; ^3^Arba Minch University, Arba Minch, Ethiopia; ^4^Department of Computer Science, Government Bikram College of Commerce, Patiala, India; ^5^All India Institute of Medical Science, Rishikesh, India

## Abstract

The correct prediction of heart disease can prevent life threats, and incorrect prediction can prove to be fatal at the same time. In this paper different machine learning algorithms and deep learning are applied to compare the results and analysis of the UCI Machine Learning Heart Disease dataset. The dataset consists of 14 main attributes used for performing the analysis. Various promising results are achieved and are validated using accuracy and confusion matrix. The dataset consists of some irrelevant features which are handled using Isolation Forest, and data are also normalized for getting better results. And how this study can be combined with some multimedia technology like mobile devices is also discussed. Using deep learning approach, 94.2% accuracy was obtained.

## 1. Introduction

Heart disease describes a range of conditions that affect your heart. Today, cardiovascular diseases are the leading cause of death worldwide with 17.9 million deaths annually, as per the World Health Organization reports [1]. Various unhealthy activities are the reason for the increase in the risk of heart disease like high cholesterol, obesity, increase in triglycerides levels, hypertension, etc. [1]. There are certain signs which the American Heart Association [2] lists like the persons having sleep issues, a certain increase and decrease in heart rate (irregular heartbeat), swollen legs, and in some cases weight gain occurring quite fast; it can be 1-2 kg daily [3]. All these symptoms resemble different diseases also like it occurs in the aging persons, so it becomes a difficult task to get a correct diagnosis, which results in fatality in near future.

But as time is passing, a lot of research data and patients records of hospitals are available. There are many open sources for accessing the patient's records and researches can be conducted so that various computer technologies could be used for doing the correct diagnosis of the patients and detect this disease to stop it from becoming fatal. Nowadays it is well known that machine learning and artificial intelligence are playing a huge role in the medical industry. We can use different machine learning and deep learning models to diagnose the disease and classify or predict the results. A complete genomic data analysis can easily be done using machine learning models. Models can be trained for knowledge pandemic predictions and also medical records can be transformed and analyzed more deeply for better predictions [4–6].

Many studies have been performed and various machine learning models are used for doing the classification and prediction for the diagnosis of heart disease. An automatic classifier for detecting congestive heart failure shows the patients at high risk and the patients at low risk by Melillo et al. [7]; they used machine learning algorithm as CART which stands for Classification and Regression in which sensitivity is achieved as 93.3 percent and specificity is achieved as 63.5 percent. Then for improving the performance electrocardiogram (ECG) approach is suggested by Rahhal et al. [8] in which deep neural networks are used for choosing the best features and then using them. Then, for detecting heart failures, a clinical decision support system is contributed by Guidi et al. [9] for preventing it at an early stage. They tried to compare different machine learning models and deep learning models especially neural networks, as support vector machine, random forest, and CART algorithms. An 87.6 percent accuracy was achieved by random forest and CART, which outperformed everyone used in the classification. Combining the natural language processing with the rule-based approach, Zhang et al. [10] achieved 93.37 percent accuracy when the NYHA HF class was found from the unstructured clinical notes. SVM techniques used for detecting patients who already have diabetes and then predicting heart disease by Parthiban and Srivatsa [11] achieved a 94.60 percent accuracy rate, and the features taken were common like blood sugar level, age of the patient, and their blood pressure data.

In machine learning, a common problem is the high dimensionality of the data; the datasets which we use contain huge data and sometimes we cannot view that data even in 3D, which is also called the curse of dimensionality [12]. So, when we perform operations on this data, we require a huge amount of memory, and sometimes the data can also grow exponentially and overfitting can happen. The weighting features can be used, so the redundancy in the dataset can be decreased which in turn also helps in decreasing the processing time of the execution [13–17]. For decreasing the dimensionality of the dataset, there are various feature engineering and feature selection techniques which can be used to remove that data not having that much importance in the dataset [18].

In literature, when feature engineering and feature selection are applied, the results improve, both for classification as well as predictions. Dun et al. [19] tried various machine learning and deep learning techniques for detecting the heart disease and also performed hyperparameters tuning for increasing the results accuracy. Neural networks achieved high accuracy of 78.3 percent, and the other models were logistic regression, SVM, and ensemble techniques like Random Forest, etc. For reducing the cardiovascular features, Singh et al. [20] used generalized discriminant analysis for extracting nonlinear features; a binary classifier like an extreme learning machine for less overfitting and increasing the training speed and the ranking method used for all these was Fisher. The accuracy achieved was 100 percent for detecting coronary heart disease. Arrhythmias classification was done by Yaghouby et al. [21] for heart rate variability. A multilayer perceptron neural network was used for doing the classification and 100 percent accuracy is achieved by reducing the features or Gaussian Discriminant Analysis. Asl et al. [22] used Gaussian discriminant analysis for reducing the HRV signal features to 15 and 100 percent precision is achieved using the SVM classifier.

For dealing with data that are of high variance or high dimensional data, by using appropriate dimensionality reduction techniques like PCA, we can store valuable information in new components [23]. PCA is used by many researchers as the first preference while dealing with high dimensionality data. Rajagopal and Ranganathan [24] used five different dimensionality reduction techniques which are unsupervised (linear and nonlinear), and neural network is used as a classifier for classifying cardiac arrhythmia. FastICA (used for independent component analysis) with a minimum of 10 components was able to achieve an F1 score of 99.83 percent. Zhang et al. [25] used the AdaBoost algorithm which is based on PCA for detecting breast cancer. Negi et al. [26] combined uncorrelated discriminant analysis with PCA so that the best features that are used for controlling the upper limb motions can be selected and the results were great. Avendaño-Valencia et al. [27] tried to reduce heart sounds to increase performance by applying PCA techniques on time-frequency representations. Kamencay et al. [28] tried a new method for different medical images reaching an accuracy of 83.6 percent when trained on 200 images by using PCA-KNN which is a scale-invariant feature used in medical images for the scaling purpose. Ratnasari et al. [29] used a gray-level threshold of 150 based on PCA and ROI, all of these used for reducing features of the X-ray images.

The studies of the past are mainly based on a 13-feature dataset. The classification is common in every study to predict if a patient has heart disease or not, and also one most common pattern which can be seen is that the dataset commonly used is of Cleveland [30]. The results obtained achieved great accuracies like random forest with 89.2 percent accuracy [31]; decision tree with 89.1 percent accuracy [32]; ANN with 92.7 percent accuracy [33], 89 percent [33], and 89.7 percent accuracy [34]; and SVM accuracy with 88 percent [34]. A hybrid model is created which achieved an accuracy of 94.2 percent by GA þ NN [35]. PCA models achieved an accuracy of 92 and 95.2 percent as PCA þ regression and PCA1þNN [36]. The dimensionality reduction was the main focus here for learning three things: (i) selection of the best features, (ii) validation of performance, and (iii) use of six different classifiers for calculating the 74 features which are selected.

Heart disease is very fatal and it should not be taken lightly. Heart disease happens more in males than females, which can be read further from Harvard Health Publishing [37]. Researchers found that, throughout life, men were about twice as likely as women to have a heart attack. That higher risk persisted even after they accounted for traditional risk factors of heart disease, including high cholesterol, high blood pressure, diabetes, body mass index, and physical activity. The researchers are working on this dataset as it contains certain important parameters like dates from 1998, and it is considered as one of the benchmark datasets when someone is working on heart disease prediction. This dataset dates from 1988 and consists of four databases: Cleveland, Hungary, Switzerland, and Long Beach V, and the results achieved are quite promising.

The rest of the paper is divided into four sections.  Section 1 consists of the introduction, Section 2 consists of the literature review, Section 3 consists of the methodology used, Section 4 consists of the discussion, Section 4 consists of the results analysis, and Section 5 consists of conclusion and future scope.

## 2. Literature Review

The summary of the literature review can be seen in Table 1. Several approaches have been performed on this popular dataset, but the accuracy obtained by all the approaches is more with time computations.

## 3. Methodology

### 3.1. Description of the Dataset

The dataset used for this research purpose was the Public Health Dataset and it is dating from 1988 and consists of four databases: Cleveland, Hungary, Switzerland, and Long Beach V. It contains 76 attributes, including the predicted attribute, but all published experiments refer to using a subset of 14 of them. The “target” field refers to the presence of heart disease in the patient. It is integer-valued 0 = no disease and 1 = disease. The first four rows and all the dataset features are shown in Table 1 without any preprocessing. Now the attributes which are used in this research purpose are described as follows and for what they are used or resemble:

- Age—age of patient in years, sex—(1 = male; 0 = female).
- Cp—chest pain type.
- Trestbps—resting blood pressure (in mm Hg on admission to the hospital). The normal range is 120/80 (if you have a normal blood pressure reading, it is fine, but if it is a little higher than it should be, you should try to lower it. Make healthy changes to your lifestyle).
- Chol—serum cholesterol shows the amount of triglycerides present. Triglycerides are another lipid that can be measured in the blood. It should be less than 170 mg/dL (may differ in different Labs).
- Fbs—fasting blood sugar larger than 120 mg/dl (1 true). Less than 100 mg/dL (5.6 mmol/L) is normal, and 100 to 125 mg/dL (5.6 to 6.9 mmol/L) is considered prediabetes.
- Restecg—resting electrocardiographic results.
- Thalach—maximum heart rate achieved. The maximum heart rate is 220 minus your age.
- Exang—exercise-induced angina (1 yes). Angina is a type of chest pain caused by reduced blood flow to the heart. Angina is a symptom of coronary artery disease.
- Oldpeak—ST depression induced by exercise relative to rest.
- Slope—the slope of the peak exercise ST segment.
- Ca—number of major vessels (0–3) colored by fluoroscopy.
- Thal—no explanation provided, but probably thalassemia (3 normal; 6 fixed defects; 7 reversible defects).
- Target (T)—no disease = 0 and disease = 1, (angiographic disease status).

### 3.2. Preprocessing of the Dataset

The dataset does not have any null values. But many outliers needed to be handled properly, and also the dataset is not properly distributed. Two approaches were used. One without outliers and feature selection process and directly applying the data to the machine learning algorithms, and the results which were achieved were not promising. But after using the normal distribution of dataset for overcoming the overfitting problem and then applying Isolation Forest for the outlier's detection, the results achieved are quite promising. Various plotting techniques were used for checking the skewness of the data, outlier detection, and the distribution of the data. All these preprocessing techniques play an important role when passing the data for classification or prediction purposes.

#### 3.2.1. Checking the Distribution of the Data

The distribution of the data plays an important role when the prediction or classification of a problem is to be done. We see that the heart disease occurred 54.46% of the time in the dataset, whilst 45.54% was the no heart disease. So, we need to balance the dataset or otherwise it might get overfit. This will help the model to find a pattern in the dataset that contributes to heart disease and which does not as shown in Figure 1.

#### 3.2.2. Checking the Skewness of the Data

For checking the attribute values and determining the skewness of the data (the asymmetry of a distribution), many distribution plots are plotted so that some interpretation of the data can be seen. Different plots are shown, so an overview of the data could be analyzed. The distribution of age and sex, the distribution of chest pain and trestbps, the distribution of cholesterol and fasting blood, the distribution of ecg resting electrode and thalach, the distribution of exang and oldpeak, the distribution of slope and ca, and the distribution of thal and target all are analyzed and the conclusion is drawn as shown in Figures 2 and 3.

By analyzing the distribution plots, it is visible that thal and fasting blood sugar is not uniformly distributed and they needed to be handled; otherwise, it will result in overfitting or underfitting of the data.

#### 3.2.3. Checking Stats of the Normal Distribution of Data

Checking the features which are important for heart disease and not important for heart disease is shown in Figures 4 and 5, respectively. Here the important factors show a different variation which means it is important.

The conclusion which can be drawn from these statistical figures is that we can see a Gaussian distribution which is important for heart disease and no Gaussian distribution which is playing that much important role in heart disease.

#### 3.2.4. Feature Selection

For selecting the features and only choosing the important feature, the Lasso algorithm is used which is a part of embedded methods while performing feature selection. It shows better predictive accuracy than filter methods. It renders good feature subsets for the used algorithm. And then for selecting the selected features, select from the model which is a part of feature selection in the scikit-learn library.

#### 3.2.5. Checking Duplicate Values in the Data

The duplicates should be tackled down safely or otherwise would affect the generalization of the model. There might be a chance if duplicates are not dealt with properly; they might show up in the test dataset which is also in the training dataset. The duplicate values can be seen in Table 2.

### 3.3. Machine Learning Classifiers Proposed

The proposed approach was applied to the dataset in which firstly the dataset was properly analyzed and then different machine learning algorithms consisting of linear model selection in which Logistic Regression was used. For focusing on neighbor selection technique KNeighborsClassifier was used, then tree-based technique like DecisionTreeClassifier was used, and then a very popular and most popular technique of ensemble methods RandomForestClassifier was used. Also for checking the high dimensionality of the data and handling it, Support Vector Machine was used. Another approach which also works on ensemble method and Decision Tree method combination is XGBoost classifier as shown in Figures 6 and 7.

### 3.4. Deep Learning Pseudocode

- Dataset of training
- Dataset of testing
- Checking the shape/features of the input
- The procedure of initiating the sequential layer
- Adding dense layers with dropout layers and ReLU activation functions
- Adding a last dense layer with one output and binary activation function
- End repeat
- L (output)
- End procedure

### 3.5. Deep Learning Proposed

There are two ways a deep learning approach can be applied. One is using a sequential model and another is a functional deep learning approach. In this particular research, the first one is used. A sequential model with a fully connected dense layer is used, with the flatten and dropout layers to prevent the overfitting and the results are compared of the machine learning and deep learning and variations in the learning including computational time and accuracy can be analyzed and can be seen in the figures further discussed in the Results section.

### 3.6. Evaluation Process Used

For the evaluation process, confusion matrix, accuracy score, precision, recall, sensitivity, and F1 score are used. A confusion matrix is a table-like structure in which there are true values and predicted values, called true positive and true negative. It is defined in four parts: the first one is true positive (TP) in which the values are identified as true and, in reality, it was true also. The second one is false positive (FP) in which the values identified are false but are identified as true. The third one is false negative (FN) in which the value was true but was identified as negative. The fourth one is true negative (TN) in which the value was negative and was truly identified as negative. The table is shown in Figure 8.

In Figure 8, P = positive, N = negative, TP = true positive, FN = false negative, FP = false positive, TN = true negative.

Then for checking how well a model is performing, an accuracy score is used. It is defined as the true positive values plus true negative values divided by true positive plus true negative plus false positive plus false negative. The formula is

(1) $$\begin{array}{c} \text{accuracy}=\frac{\text{ TP}+\text{ TN}}{\text{TP}+\text{TN}+\text{FP}+\text{FN}}. \end{array}$$

After accuracy there is specificity which is the proportion of true negative cases that were classified as negative; thus, it is a measure of how well a classifier identifies negative cases. It is also known as the true negative rate. The formula is

(2) $$\begin{array}{c} \text{specificity}=\frac{\text{TN}}{\text{TN}+\text{FP}}. \end{array}$$

Then there is sensitivity in which the proportion of actual positive cases got predicted as positive (or true positive). Sensitivity is also termed as recall. In other words, an unhealthy person got predicted as unhealthy. The formula is

(3) $$\begin{array}{c} \text{sensitivity}=\frac{\text{TP}}{\text{TP}+\text{FN}}. \end{array}$$

### 3.7. Use of Multimedia

The whole knowledge which will be obtained could be transferred to the mobile devices means, when the person will input these symptoms in the mobile device in which the trained model will already be present and then can analyze the symptoms and could give the prescription accordingly. Different doctors could be taken under consideration and a complete autonomous system could be generated. We can also integrate the doctors' numbers if the model is showing high risk and they can consult the doctor. And if they are showing less symptoms, then medicines already prescribed by the doctors for a certain range will be shown. This system will prove beneficial and the workload on the doctors would also be less. Also in these current times of coronavirus, we need more autonomous systems which would also help in keeping the virtuality between persons more. Thus we could create some applications with the help of doctors and make it work.

## 4. Analysis of Results

By applying different machine learning algorithms and then using deep learning to see what difference comes when it is applied to the data, three approaches were used. In the first approach, normal dataset which is acquired is directly used for classification, and in the second approach, the data with feature selection are taken care of and there is no outliers detection. The results which are achieved are quite promising and then in the third approach the dataset was normalized taking care of the outliers and feature selection; the results achieved are much better than the previous techniques, and when compared with other research accuracies, our results are quite promising.

### 4.1. Using the First Approach (without Doing Feature Selection and Outliers Detection)

As can be seen in Figure 1, the dataset is not normalized, there is no equal distribution of the target class, it can further be seen when a correlation heatmap is plotted, and there are so many negative values; it can be visualized in Figure 9.

So, even if the feature selection is done, still, we have outliers which can be seen in Figure 10.

By applying the first approach, the accuracy achieved by the Random Forest is 76.7%, Logistic Regression is 83.64%, KNeighbors is 82.27%, Support Vector Machine is 84.09%, Decision Tree is 75.0%, and XGBoost is 70.0%. SVM is having the highest accuracy here which is achieved by using the cross-validation and grid search for finding the best parameters or in other words doing the hyperparameter tuning. Then after machine learning, deep learning is applied by using the sequential model approach. In the model, 128 neurons are used and the activation function used is ReLU, and in the output layer which is a single class prediction problem, the sigmoid activation function is used, with loss as binary cross-entropy and gradient descent optimizer as Adam. The accuracy achieved is 76.7%.

### 4.2. Using the Second Approach (Doing Feature Selection and No Outliers Detection)

After selecting the features (feature selection) and scaling the data as there are outliers, the robust standard scalar is used; it is used when the dataset is having certain outliers. In the second approach, the accuracy achieved by Random Forest is 88%, the Logistic Regression is 85.9%, KNeighbors is 79.69%, Support Vector Machine is 84.26%, the Decision Tree is 76.35%, and XGBoost is 71.1%. Here the Random Forest is the clear winner with a precision of 88.4% and an F1 score of 86.5%.

Then deep learning is applied with the same parameters before and the accuracy achieved is 86.8%, and the evaluation accuracy is 81.9%, which is better than the first approach.

### 4.3. Using the Third Approach (by Doing Feature Selection and Also Outliers Detection)

In this approach, the dataset is normalized and the feature selection is done and also the outliers are handled using the Isolation Forest. The correlation comparison can be seen in Figure 10. The accuracy of the Random Forest is 80.3%, Logistic Regression is 83.31%, KNeighbors is 84.86%, Support Vector Machine is 83.29%, Decision Tree is 82.33%, and XGBoost is 71.4%. Here the winner is KNeighbors with a precision of 77.7% and a specificity of 80%. A lot of tips and tricks for selecting different algorithms are shown by Garate-Escamila et al. [38]. Using deep learning in the third approach, the accuracy achieved is 94.2%. So, the maximum accuracy achieved by the machine learning model is KNeighbors ( 83.29%) in the third approach, and, for deep learning, the maximum accuracy achieved is 81.9%. Thus, the conclusion can be drawn here that, for this dataset, the deep learning algorithm achieved 94.2 percent accuracy which is greater than the machine learning models. We also made a comparison with another research of the deep learning by Ramprakash et al. [39] in which they achieved 84% accuracy and Das et al. [33] achieved 92.7 percent accuracy. So our algorithm produced greater accuracy and more promising than other approaches [40, 41]. The comparison of different classifiers of ML and DL can be seen in Table 3.

### 4.4. Architecture for Using Deep Learning Approach

Here in this architecture, we used three dense layers: the first dense layer consists of 128 units, the second dense layer consists of 64 units, and the third dense layer consists of 32 units. For the first layer, the Dropout Layer (HyperParameter) is 0.2 and for the second is 0.1.

## 5. Conclusion and Future Scope

In this paper, we proposed three methods in which comparative analysis was done and promising results were achieved. The conclusion which we found is that machine learning algorithms performed better in this analysis. Many researchers have previously suggested that we should use ML where the dataset is not that large, which is proved in this paper. The methods which are used for comparison are confusion matrix, precision, specificity, sensitivity, and F1 score. For the 13 features which were in the dataset, KNeighbors classifier performed better in the ML approach when data preprocessing is applied.

The computational time was also reduced which is helpful when deploying a model. It was also found out that the dataset should be normalized; otherwise, the training model gets overfitted sometimes and the accuracy achieved is not sufficient when a model is evaluated for real-world data problems which can vary drastically to the dataset on which the model was trained. It was also found out that the statistical analysis is also important when a dataset is analyzed and it should have a Gaussian distribution, and then the outlier's detection is also important and a technique known as Isolation Forest is used for handling this. The difficulty which came here is that the sample size of the dataset is not large. If a large dataset is present, the results can increase very much in deep learning and ML as well. The algorithm applied by us in ANN architecture increased the accuracy which we compared with the different researchers. The dataset size can be increased and then deep learning with various other optimizations can be used and more promising results can be achieved. Machine learning and various other optimization techniques can also be used so that the evaluation results can again be increased. More different ways of normalizing the data can be used and the results can be compared. And more ways could be found where we could integrate heart-disease-trained ML and DL models with certain multimedia for the ease of patients and doctors.

## Figures and Tables

**Figure 1:** Class distribution of disease and no disease.

**Figure 2:** Distribution of age and sex.

**Figure 3:** Distribution of chest pain and trestbps.

**Figure 4:** Features important for heart disease.

**Figure 5:** Features not important for heart disease.

**Figure 6:** 1st schematic diagram of the proposed model.

**Figure 7:** 2nd schematic diagram of the proposed model.

**Figure 8:** Confusion matrix.

**Figure 9:** Correlation heatmap.

**Figure 10:** Feature selection on correlation heatmap.

**Table 1:** Summary of the literature review.

Sr.no.	Author	Year	Findings
1	Gárate-Escamila et al. [38]	2020	DNN and ANN were used with the X ^ 2 statistical model. The clinical data parameters were used for conforming the predictions.
2	Harvard Medical School [37]	2020	Hungarian-Cleveland datasets were used for predicting heart disease using different machine learning classifiers and PCA was used for dimensionality reduction and feature selection
3	Zhang et al. [25]	2018	AdaBoost classifier with PCA combination was used for the feature extraction and the accuracy of the prediction was increased
4	Singh et al. [20]	2018	Heart rate variability was for the detection of coronary artery disease. Fisher method and generalised discriminant analysis with binary classifiers were used for the detection of important features.
5	Chen et al. [16]	2018	A subspace feature clustering was used as a subset of stratified feature clustering and for doing a feature reduction of the clusters formed
6	Yang and Nataliani [15]	2018	A fuzzy clustering method especially fuzzy c-means was used for various feature weighted methods and features were reduced
7	Kumar [32]	2017	Different machine learning algorithms were applied for getting the results and then compared with each other
8	Rajagopal and Ranganathan [24]	2017	Combination of probabilistic neural network classifier, PCA, kernel PCA, and unsupervised dimensionality reduction was used so that feature reduction can be used and a domain expert was used for the correct analysis of the result
9	Zhang et al. [10]	2017	Support vector machine is used for the classification purpose of the clinical data which is matched with the codes of New York heart association; further findings are left for other researchers
10	Khan and Quadri [31]	2016	The main aim of this research was to summarize the best model and angiographic disease status by analyzing different unstructured data and using data mining techniques
11	Negi et al. [26]	2016	Uncorrelated linear discriminant analysis with PCA was used for studying the electrocardiogram and Wilson methods were also used for the distinction of upper limb motions
12	Dun et al. [19]	2016	They applied a variety of deep learning techniques and ensemble techniques and also performed hyperparameter tuning techniques for increasing the accuracy.
13	Rahhal et al. [8]	2016	ECG approach is used by consulting various domain experts and then MIT-BIH arrhythmia database as well as two other databases called INCART and SVDB, respectively
14	Imani and Ghassemian [17]	2015	There are several times when the data is not enough, so Imani approached a weighted training sample method including feature extraction for the spatial dimension of the images and the accuracy was increased
15	Guidi et al. [9]	2014	Neural networks, SVM, and fuzzy system approach are used and Random Forest is used as a classifier, for the prediction of heart failure by using a clinical decision support system
16	Santhanam and Ephzibah [36]	2013	A regression technique with PCA with its different versions like PCA1, PCA2, PCA3, and PCA4 was used and the features were extracted and the results were promising
17	Ratnasari et al. [29]	2013	The datasets used were Cleveland–Hungarian dataset and the UCI machine learning datasets were analyzed with feature selection techniques
18	Kamencay et al. [28]	2013	Object recognition was performed with scale-invariant feature transformation. Caltech 101 database was used for the evaluation purpose.
19	Melillo et al. [7]	2013	Two public Holster databases were used for finding high-risk and low-risk patients. Cart algorithm is applied for the classification purpose.
20	Amma [35]	2012	The dataset used was from University of California, Irvine. The genetic algorithm was used for the training purpose and neural network for the classification purpose.
21	Keogh and Mueen [12]	2012	How to break the curse of dimensionality using PCA, SVM, and other classifiers and reduce features.
22	Parthiban and Srivatsa [11]	2012	Diabetes is one of the main causes of heart disease. The classifiers used are Naïve Bayes and SVM for extracting important features and classification purpose.
23	Srinivas et al. [34]	2010	Prediction of heart diseases in the coal mines was the prime consideration, and decision tree, naïve Bayes, and neural networks were used for the classification
24	Das et al. [33]	2009	On Cleveland dataset, using a SAS-based software, a great accuracy was achieved with different ensemble techniques
25	Yaghouby et al. [21]	2009	Cardiac arrhythmias was considered using the MIT-BIH database. HRV similar to [20] was used.
26	Asl et al. [22]	2008	Generalised discriminant analysis and SVM were used for feature reduction and classification
27	Avendaño-Valencia et al. [27]	2009	Feature extraction was based upon the heart murmur frequency with time representation frequency and PCA was used for the analysis of the features
28	Guyon et al. [23]	2008	Book for doing feature extraction efficiently.
29	UCI Machine Learning Repository [30]	1998	This dataset is used for many ML and deep learning benchmark results
30	Liu and Motoda [18]	1998	Feature importance and how to select them appropriately was discussed in this book
31	Wettschereck et al. [14]	1997	K-NN algorithm was used for the classification as they are mostly the derivatives for the lazy learning algorithms for the feature selection using weighted methods
32	Wettschereck and Dietterich [13]	1995	Different classification problems decision boundaries were analyzed, and the problem was tackled using nested generalized example

**Table 2:** Duplicate values.

Age	Sex	Cp	Trest bps	Chol	Rest ecg	Thalach	Exang	Old peak	Slope	Ca	Thal	T
38	1	2	138	175	1	173	0	0.0	2	4	2	1

Using the pandas' function for dropping these values is the simplest. It is also an important part while performing data preprocessing.

**Table 3:** Comparative analysis.

Classifiers	Accuracy (%)	Specificity	Sensitivity
Logistic regression	83.3	82.3	86.3
K neighbors	84.8	77.7	85.0
SVM	83.2	78.7	78.2
Random forest	80.3	78.7	78.2
Decision tree	82.3	78.9	78.5
DL	94.2	83.1	82.3

## Data Availability

The data used to support the findings of this study are available from the corresponding author upon request.
